# The Effect of Different Nutritional Nursing Support on the Nutritional Status and Disease Recovery of Elderly Patients with Gastrointestinal Tumors during the Perioperative Period

**DOI:** 10.1155/2022/4977922

**Published:** 2022-06-29

**Authors:** Lingzhi Chen, Sixin Zheng, Qi Xie, Liping Huang, Guang Yin

**Affiliations:** Department of Gastrointestinal Surgery, Affiliated Hangzhou First People's Hospital, Zhejiang University School of Medicine, 310006 Hangzhou, China

## Abstract

**Objective:**

This study explored the effect of different nutritional nursing support on nutritional status, immune function, postoperative bowel motility, and complications in elderly patients with gastrointestinal tumors during the perioperative period.

**Methods:**

300 patients with gastrointestinal tumors treated in the Department of Gastroenterology and anorectal surgery of Hangzhou First People's Hospital Affiliated with the Medical College of Zhejiang University from February 2018 to March 2020 were selected as the research objects in this study. Patients were divided into the early enteral nutrition (EEN) and total parenteral nutrition (TPN) groups (150 cases in each group) according to the principle of odd and even admission numbers. The patients in the EEN and TPN groups were given enteral nutrition nursing support and parenteral nutrition nursing support, respectively. The nutritional status, immune function, postoperative bowel motility, and complication rate of the two groups were evaluated 7 days after the operation.

**Results:**

The nutritional indexes decreased 3 days after the operation and gradually recovered 7 days after the operation in both groups with different nutritional nursing support. The Hb, TRF, PAB, and ALB indexes in the TPN group were significantly lower than those in the EEN group (*P* < 0.01). On the 7th day after the operation, the indexes of peripheral blood immunoglobulin (IgG, IgM, and IgA) were significantly lower than those in the TPN group, and T lymphocyte subsets (CD4, CD8, and CD4/CD8) demonstrated that the immunological indexes of patients in the EEN group were significantly higher than those in the TPN group (*P* < 0.01). In terms of intestinal peristalsis, the time of first exhaust and first defecation in the EEN group was significantly shorter than that in the TPN group (*P* < 0.01) during the perioperative period. Furthermore, both groups had different degrees of complications, while patients demonstrated a lower complication rate in the EEN group compared to those in the TPN group, suggesting a safer postoperative mode. The results of subgroup analysis showed that the nutritional indexes of the gastric cancer group 7 days after operation were significantly higher than those of the colorectal cancer group under EEN and TPN nutritional support modes.

**Conclusion:**

Clinical results have suggested that enteral nutrition nursing support can improve the perioperative nutritional status of elderly patients with gastrointestinal tumors by enhancing the immune function and promoting intestinal peristalsis. Meanwhile, the postoperative EEN mode reduces the rate of complications and demonstrates higher safety. Therefore, it has a high clinical application value.

## 1. Introduction

Gastrointestinal cancer is one of the incidence rates of malignant tumors. Gastrointestinal cancer leads to different effects on the digestive and metabolic functions of the body due to its relatively special location. Therefore, malnutrition and low immune function are commonly seen in gastrointestinal cancer patients, especially the elderly [1, 2]. Relevant studies have shown that postoperative malnutrition can lead to wound infection, abdominal infection, anastomotic fistula, pulmonary dysfunction, poor postoperative wound healing, and other complications [3, 4]. In addition, the stress caused by surgical treatment of gastrointestinal tumors can lead to systemic inflammatory reactions, which severely impact the prognosis. Therefore, giving necessary early nutritional support and related nursing methods to patients with gastrointestinal tumors after the operation is of great significance to reduce the incidence of postoperative complications, enhance the body's resistance and immunity, improve the nutritional status of patients, and promote the early healing of postoperative incision [5, 6]. At present, total parenteral nutrition (TPN) and early enteral nutrition (EEN) are the two standard nutritional nursing support after gastrointestinal tumor operation. However, it is essential to explore how to minimize the burden and adverse reactions of the digestive tract and promote the effective absorption and utilization of nutrients during the process of nutritional nursing support. There were many studies on perioperative nutritional support for gastrointestinal tumors [7, 8]. The results illustrated that enteral nutrition support was more helpful than parenteral nutrition to improve the nutritional status and immune capacity of patients, thus reducing postoperative complications of the disease and improving patient outcomes. However, relevant studies are limited to older age groups and are mostly limited to random cross-sectional observations. This comparative study evaluates the effects of TPN and EEN nutritional nursing support in elderly patients with gastrointestinal tumors by examining perioperative nutritional status, immune function, postoperative bowel motility, and complications of patients during the perioperative period.

## 2. Materials and Methods

### 2.1. Objects and Groups

In this study, 300 elderly patients with gastrointestinal tumors treated in the Department of Gastrointestinal and Anal Surgery of Hangzhou First People's Hospital Affiliated with the Medical College of Zhejiang University from February 2018 to March 2020 were selected as the research objects. The flowchart is shown in Figure 1. All subjects were diagnosed with gastric cancer, colon cancer, and rectal cancer by pathological [9] examination and received radical surgical treatment. Patients were divided into the EEN and TPN groups (150 cases in each group) according to the single and double mantissa of admission numbers in this study. There was no significant difference in general data (such as gender, age, and tumor type) between the two groups (*P* > 0.05), which was in line with the conditions of the clinical control study. This study has been reported to the hospital ethics committee for review and approval. Inclusion criteria include (1) patients with primary gastrointestinal tumor confirmed by clinicopathological diagnosis; (2) patients receiving radical surgical treatment; (3) no serious organic lesions in the crucial organs and no other diseases such as blood, immunity, metabolism, and infectious diseases; (4) no mental disorder or cognitive impairment; (5) ability to well tolerate nutritional support methods used in this study and to complete the whole research process; and (6) voluntary participation of patients and their families in the study and signed informed consent when they knew the purpose, methods, and risks of the study. Exclusion criteria include (1) patients with malignant tumor metastasis or other types of tumor diseases, (2) patients receiving palliative resection, (3) complication of organic lesions of important organs, and (4) those who cannot stand the nutritional support approach adopted in the study or who cannot complete the whole research process.

### 2.2. Nursing Methods

For the TPN group, patients in this group were treated with total parenteral nutrition. For the specific methods, on the first day after the operation, the nutrients required by the body, including glucose, electrolyte, compound amino acids, fat emulsion, water-soluble vitamins, fat-soluble vitamins, trace elements, and other nutrients, were prepared according to the doctor's advice and put into 3 L bags in an all-in-one form. Nutritional support was implemented by intravenous drip. The daily nutrient supply should be controlled at 25-35 kcal/kg, and the daily infusion time should be controlled at 18 h~24 h. During the treatment, the proportion and amount of nutrients were reasonably adjusted according to the biochemical blood test results. All patients were given parenteral venous nutritional support for one week. After the operation, a liquid diet could be given transiently according to the recovery of gastrointestinal function. For the EEN group, the patients in this group were cared for by early enteral nutrition support. For the specific method, the nasal intestinal tube into the operation was placed, and the position should be able to reach about 25 cm below the trochanter ligament or jejunal output loop. On the first day after the operation, 250 mL of 9% normal saline was slowly input through the nasal intestinal tube. The dropping rate should be controlled at 20 mL/h. During enteral nutrition support, the vital signs of the patient should be closely observed. If the patient does not feel any discomfort, the dropping rate can be appropriately accelerated. On the second day after the operation, 200 mL enteral nutrition emulsion (provided by Huarui Pharmaceutical Co., Ltd., 200 mL/bottle, H20040722)+5% glucose solution can be given. The initial dropping rate should be controlled at 25 mL/h, and the maximum rate should be controlled within 125 mL/h according to the patient's tolerance every 12 h or 24 h. At the same time, a heater was used to maintain the temperature of the nutrient solution at 37-42°C to avoid causing gastrointestinal discomfort. During the nursing period, generally, the solution concentration was from low to high. The infusion and infusion speed were from slow to fast. The number of nutrient solutions for a single infusion was from less to more to strive to realize the acceptable nursing of patients. All patients were given continuous enteral nutrition support for one week, and a liquid diet could be given transiently according to the recovery of gastrointestinal function. The following matters should be paid attention to during enteral nutrition care: (1) The nasal and intestinal tubes were unobstructed and unblocked and washed regularly every day. The tubes were washed with 20 mL warm boiled water once every four hours and once every two hours if necessary. The tubes were sealed with 20 mL warm boiled water with positive pressure. (2) When the tube feeding operation was carried out, the action shall be accurate and gentle to avoid sliding out of the nasal intestinal tube; take good care of the nasal cavity, properly fix the catheter, and carefully check the depth of the catheter in each shift. (3) Pay attention to the principle of aseptic operation, keep the infusion pipeline and nutrient solution clean, and avoid pollution. (4) During the nursing operation of enteral nutrition, the bedside angle (30°~45°) should be raised appropriately to prevent adverse events such as esophageal reflux and aspiration. (5) Control the amount, temperature, and concentration of nutrient solution during infusion, and adjust to the appropriate infusion speed. (6) Observe the complications and the symptoms of diarrhea, abdominal distention, vomiting, and gastric retention. If there is any discomfort, deal with it in time. (7) For psychological intervention, patients with gastrointestinal cancer are prone to different degrees of adverse emotions (such as depression, irritability, and anxiety) due to physiological discomfort after the operation. During enteral nutrition support, the placement of the nasal intestinal tube will lead to the patient's resistance. The nursing staff should explain in detail the significance, importance, and implementation method of enteral nutrition, explain that the nutrition tube is an important guarantee for the implementation of early enteral nutrition, actively dredge and appease the patients, alleviate the patient's bad mood, and strengthen the patient's trust in the medical staff. It is helpful to improve the nursing compliance of patients.

### 2.3. Observation Index

The venous blood of the two groups was collected and analyzed through the biochemical test before the operation and 3 days and 7 days after the operation by the laboratory of our hospital. The levels of hemoglobin (Hb), transferrin (TRF), prealbumin (PAB), and serum albumin (ALB) at different stages were statistically analyzed. The venous blood of the two groups was taken before operation and 7 days after the operation to examine peripheral blood immunoglobulin (main indexes are IgG, IgM, and IgA) and T lymphocyte subsets (main indexes are CD4, CD8, and CD4/CD8). The postoperative bowel motility and complications of the two groups were observed.

### 2.4. Statistical Analysis

All statistical data of this study were recorded in Excel form, and SPSS17.0 statistical software was used for statistical analysis. Nutritional index, immunological index, intestinal peristalsis index, and other measurement data were expressed by $\bar{x}\pm s$, and the independent or paired *t*-test was performed for comparison. The counting data of postoperative complications were expressed in %, and the *χ*^2^ test was performed. There was a significant difference in the statistical data of the evaluation results between the two groups, which was expressed as *P* < 0.05/*P* < 0.01.

## 3. Results

### 3.1. Baseline Characteristics of the Two Groups

There were 81 males and 69 females in the EEN group. The age range was 60-81 years, with an average age of 64.98 ± 4.65 years. The tumor types were 63 cases of gastric cancer, 54 cases of colon cancer, and 33 cases of rectal cancer. There are 83 males and 67 females in the TPN group. The age range was 60-79 years, with an average age of 64.66 ± 4.55 years. The tumor types were 64 cases of gastric cancer, 51 cases of colon cancer, and 35 cases of rectal cancer. There was no statistical difference in baseline data (*P* > 0.05) (see Table 1).

### 3.2. Nutritional Indexes of the Two Groups

Before the operation, there was no significant difference in Hb, TRF, PAB, and ALB results between the two groups (*P* > 0.05). Three days after giving different nutritional care support, the nutritional indexes of the two groups decreased, and the nutritional indexes gradually recovered seven days after the operation. However, the biochemical test results showed that the indexes of Hb, TRF, PAB, and ALB in the TPN group were significantly lower than those in the EEN group (*P* < 0.01), which showed that the postoperative nutritional status of the EEN group was significantly improved than that of the TPN group (see Table 2 and Figure 2 for the detailed statistical data).

### 3.3. Immune Function Indexes of the Two Groups

The immunological test showed that there was no significant difference in the indexes of peripheral blood immunoglobulin (IgG, IgM, and IGA) and T lymphocyte subsets (CD4, CD8, and CD4/CD8) between the two groups before the operation, and there was no significant difference between the two groups (*P* > 0.05). The test on the 7th day after the operation showed that the immunological indexes IgG, IgM, IgA, CD4, CD8, and CD4/CD8 of patients in the EEN group were significantly better than those in the TPN group. The comparison between groups was statistically significant (*P* < 0.01), which showed that the immune function of patients in the EEN group was better than that in the TPN group (see Table 3 and Figure 3 for detailed statistical data).

### 3.4. Intestinal Peristalsis Indexes of the Two Groups

Clinical observation showed that after different nutritional nursing support interventions, patients' first postoperative exhaust and first defecation time in the EEN group were significantly shorter than those in the TPN group. The comparison between groups was statistically significant (*P* < 0.01), which showed that patients' postoperative bowel motility effect in the EEN group was better than that in the TPN group (see Table 4 and Figure 4 for detailed data).

### 3.5. Indicators of Complications in the Two Groups

After the patients in the two groups were given different nutritional care support after the operation, there were various degrees of complications. Still, the complication rate of the patients in the EEN group was significantly lower than that in the TPN group. The comparison between the groups was statistically significant (*P* < 0.01), which showed that the safety of the postoperative EEN mode in patients with gastrointestinal tumors was significantly better than that in the TPN group (see Table 5 for the detailed data).

### 3.6. Comparison of Nutritional Indicators of Gastric and Colorectal Cancer in Subgroups of the Two Groups

In order to further clarify the effect of different nutritional support methods on malignant tumors in different parts, we divided the patients into two groups of gastric cancer and colorectal cancer for analysis. The results showed that after EEN support, Hb, TRF, PAB, and ALB in the gastric cancer group were significantly higher than those in the colorectal cancer group at 7 days after operation. After TPN support, Hb, PAB, and ALB in the gastric cancer group were significantly higher than those in the colorectal cancer group on the 7th day after operation (see Table 6 for details).

## 4. Discussion

Early postoperative enteral nutrition for patients with gastrointestinal tumors is mainly through the perfusion of nutrients through the pipeline. The intestine can selectively absorb nutrients, which can significantly prevent and improve the postoperative malnutrition of patients, effectively regulate the immune function of patients, and improve the inflammatory response, which is of great significance to reduce postoperative complications [10, 11]. Specific nutrients can be perfused through EEN, which can play a certain pharmacological role and can be used as one of the later rehabilitation treatment methods. Enteral nutrition support can not only effectively stimulate the rapid secretion of digestive juice from the gastrointestinal tract, promote intestinal peristalsis, and increase the blood flow of visceral organs but also is more in line with human physiological processes [12]. Meanwhile, it retains the structure and function of intestinal mucosa to the greatest extent and protects the intestinal mucosal barrier, thus preventing or reducing entheogenic infection [13]. Relevant studies [8, 14] showed that enteral nutrition was of great significance for improving nutritional status and immunity.

The results showed that the postoperative indexes of Hb, TRF, PAB, and ALB in the EEN group were significantly better than those in the TPN group. The immunological indexes of IgG, IgM, IgA, CD4, CD8, and CD4/CD8 in the EEN group were significantly better than those in the TPN group, the first postoperative exhaust and first defecation time in the EEN group were significantly shorter than those in the TPN group, and the complication rate in the EEN group was significantly lower than that in the TPN group. Studies [15, 16] reported that giving reasonable and effective nutritional nursing support to patients with gastrointestinal tumors after the operation can significantly improve their nutritional status. In the study on the recovery of gastrointestinal mucosal immune function, Becker and others [17] suggested that enteral nutrition support could effectively promote S-IgA secretion in intestinal mucosa after gastric cancer surgery, increasing the immune barrier effect of the intestinal mucosa. In addition, nutrients can change the immune status of the body by affecting the secretion of antibodies and cytokines by immune effector cells [18]. In this study, the postoperative immune globulin levels in the EEN group were significantly higher than those in the TPN group, suggesting that enteral nutrition can better improve the immune status of patients and reduce complications such as infection, which is similar to the previous report [19]. In addition, Chen et al. [20] confirmed that the presence of an appropriate amount of arginine and other immune enhancers in enteral nutrition solutions can promote the postoperative rehabilitation of patients. Studies [21, 22] showed that enteral nutrition support for patients with gastric cancer after the operation could significantly reduce the rate of postoperative complications, especially in abdominal abscess, anastomotic fistula, and mortality, and significantly shorten the length of hospital stay. Besides, it is important to pay attention to psychological counselling which can stabilize the patient's mood, eliminate concerns, and make them actively cooperate with the treatment. The recovery of postoperative intestinal function can be promoted by adjusting the temperature and infusion speed of nutrient solution. The prevention of complications can speed up the rehabilitation process of the disease. The results of subgroup analysis showed that the nutritional indexes of the gastric cancer group 7 days after operation were significantly higher than those of the colorectal cancer group under EEN and TPN nutritional support modes, suggesting that nutritional support had a better effect on postoperative nutritional recovery of gastric cancer patients.

In conclusion, enteral nutrition nursing support can improve the perioperative nutritional status of elderly patients with gastrointestinal tumors by improving the immune function and promoting intestinal peristalsis. The reduction in the complication rate and high safety suggest that enteral nutrition nursing support has a significant value in clinical application. In clinical practice, the choice of enteral/parenteral nutrition for some patients needs to be determined according to the condition, which cannot be completely randomized. Therefore, prospective, multicenter, and fully randomized studies are needed to confirm this conclusion in the future.

## Figures and Tables

**Figure 1:** Flowchart of case grouping.

**Figure 2:** Nutritional indexes (Hb, TRF, PAB, and ALB) of the two groups. Hb of 3 and 7 days after the operation, TRF of 7 days after the operation, PAB of 7 days after the operation, and ALB of 7 days after the operation in the EEN group and the TPN group (*P* < 0.001); the rest of the differences were all *P* > 0.05.

**Figure 3:** Immune function indexes (IgG, IgM, IGA, CD4, CD8, and CD4/CD8) of the two groups. Before the operation, the difference between the EEN group and the TPN group was *P* > 0.05, and the difference between the two groups at 7 days after operation was *P* < 0.05.

**Figure 4:** Intestinal peristalsis indexes of the two groups. Compared with the EEN group ^∗∗∗^*P* < 0.001.

**Table 1:** Baseline characteristics of the two groups of patients.

Baseline data	EEN group (*n* = 150)	TPN group (*n* = 150)	*t*/*χ*^2^	*P*
Age (years)	64.98 ± 4.65	64.66 ± 4.55	0.603	0.547
Gender (male/female)	81/69	83/67	0.054	0.817
Disease duration (years)	8.01 ± 1.99	8.13 ± 3.13	0.396	0.692
BMI (kg/m^2^)	24.91 ± 1.74	25.03 ± 2.04	0.544	0.587
Tumor type				
Gastric cancer	63	64	0.152	0.927
Colon cancer	54	51		
Rectal cancer	33	35		

**(a):** 

Group	Hb (g/L)			TRF (g/L)		
	Before the operation	3 days after the operation	7 days after the operation	Before the operation	3 days after the operation	7 days after the operation
EEN group	113.3 ± 8.6	105.6 ± 7.7	121.1 ± 9.7	1.73 ± 0.41	1.67 ± 0.33	3.15 ± 0.42
TPN group	112.9 ± 8.8	100.7 ± 8.0	112.9 ± 9.3	1.74 ± 0.39	1.66 ± 0.30	2.12 ± 0.35
*t*	0.337	5.428	7.545	0.192	0.324	23.088
*P*	0.736	<0.001	<0.001	0.848	0.746	<0.001

**(b):** 

Group	PAB (mg/L)			ALB (g/L)		
	Before the operation	3 days after the operation	7 days after the operation	Before the operation	3 days after the operation	7 days after the operation
EEN group	199.4 ± 47.0	179.1 ± 57.4	232.2 ± 58.6	29.7 ± 3.3	28.4 ± 3.1	39.0 ± 4.6
TPN group	190.8 ± 46.2	178.2 ± 61.1	201.2 ± 42.5	30.4 ± 3.1	28.1 ± 2.9	31.1 ± 3.0
*t*	1.605	0.136	5.247	1.740	0.821	17.617
*P*	0.110	0.892	<0.001	0.083	0.412	<0.001

**Table 3:** Statistical analysis of immune function indexes of patients in the two groups before and after nutritional support (*n* = 150, $\bar{x}\pm s$).

Group	Detection time	IgG (g/L)	IgM (g/L)	IgA (g/L)	CD4 (%)	CD8 (%)	CD4/CD8
EEN group	Before the operation	11.15 ± 2.29	1.97 ± 0.22	1.71 ± 0.34	37.19 ± 6.03	24.09 ± 9.68	1.96 ± 1.28
	7 days after the operation	16.84 ± 2.34	2.65 ± 0.52	2.80 ± 0.53	36.14 ± 2.64	28.37 ± 10.21	1.50 ± 0.77
TPN group	Before the operation	11.26 ± 2.31	1.88 ± 0.24	1.73 ± 0.40	36.89 ± 6.51	25.25 ± 8.22	1.72 ± 1.040
	7 days after the operation	13.80 ± 1.69	2.02 ± 0.77	2.02 ± 0.27	31.15 ± 4.46	22.17 ± 8.23	1.71 ± 1.04
*t* (before the operation)		0.421	3.407	0.487	0.406	1.116	1.866
*P* (before the operation)		0.674	0.001	0.627	0.685	0.266	0.063
*t* (7 days after the operation)		12.876	8.274	16.137	11.783	5.784	2.005
*P* (7 days after the operation)		<0.001	<0.001	<0.001	<0.001	<0.001	0.046

**Table 4:** Statistical analysis of intestinal peristalsis indexes of patients in the two groups after nutritional support (*n* = 150, $\bar{x}\pm s$, d).

Group	First postoperative exhaust time	First defecation time after operation
EEN group	2.12 ± 0.76	3.07 ± 0.81
TPN group	3.34 ± 0.89	5.36 ± 1.32
*t*	12.785	18.099
*P*	<0.001	<0.001

**Table 5:** Statistical analysis of complication indexes of patients in the two groups after nutritional support (*n* = 150, *n* (%)).

Group	Incision infection	Abdominal infection	Pneumonia	Anastomotic fistula	Stomach discomfort	Complication rate
EEN group	4 (2.67)	4 (2.67)	4 (2.67)	0	14 (9.33)	26 (17.34)
TPN group	13 (8.67)	8 (5.33)	9 (6)	15 (10)	22 (14.67)	67 (44.67)
*χ* ^2^	5.051	1.389	2.010	15.790	2.020	26.196
*P*	0.025	0.239	0.156	<0.001	0.155	<0.001

**(a):** 

Group	Hb (g/L)			TRF (g/L)		
	Before the operation	3 days after the operation	7 days after the operation	Before the operation	3 days after the operation	7 days after the operation
Gastric cancer EEN group	112.6 ± 9.6	107.6 ± 7.0	123.6 ± 8.9	1.71 ± 0.46	1.65 ± 0.33	3.24 ± 0.40
Colorectal cancer EEN group	113.9 ± 7.5	103.8 ± 8.0	118.7 ± 9.9	1.76 ± 0.36	1.70 ± 0.33	3.06 ± 0.43
*t*	-0.858	3.080	3.176	-0.731	-0.929	2.680
*P*	0.391	0.003	0.002	0.464	0.355	0.008

**(b):** 

Group	PAB (mg/L)			ALB (g/L)		
	Before the operation	3 days after the operation	7 days after the operation	Before the operation	3 days after the operation	7 days after the operation
Gastric cancer EEN group	202.4 ± 47.1	181.7 ± 61.2	247.6 ± 52.2	29.4 ± 3.7	28.6 ± 3.0	40.1 ± 4.1
Colorectal cancer EEN group	196.5 ± 47.0	176.6 ± 53.8	217.3 ± 60.8	30.0 ± 2.8	28.2 ± 3.2	38.0 ± 4.8
*t*	0.772	0.543	3.274	-1.041	0.733	2.914
*P*	0.441	0.587	0.001	0.298	0.465	0.004

**(c):** 

Group	Hb (g/L)			TRF (g/L)		
	Before the operation	3 days after the operation	7 days after the operation	Before the operation	3 days after the operation	7 days after the operation
Gastric cancer EEN group	113.3 ± 7.7	101.4 ± 8.2	115.0 ± 9.1	1.78 ± 0.41	1.64 ± 0.28	2.16 ± 0.32
Colorectal cancer EEN group	112.5 ± 9.9	100.1 ± 7.8	110.7 ± 9.1	1.70 ± 0.36	1.67 ± 0.32	2.08 ± 0.38
*t*	0.592	1.052	2.888	1.271	-0.590	1.440
*P*	0.555	0.295	0.004	0.206	0.556	0.152

**(d):** 

Group	PLB (g/L)			ALB (g/L)		
	Before the operation	3 days after the operation	7 days after the operation	Before the operation	3 days after the operation	7 days after the operation
Gastric cancer EEN group	188.1 ± 47.7	173.1 ± 63.2	210.8 ± 41.3	30.5 ± 3.2	27.9 ± 3.1	31.7 ± 2.9
Colorectal cancer EEN group	193.5 ± 44.8	183.3 ± 58.8	191.7 ± 41.8	30.3 ± 3.0	28.3 ± 2.6	30.6 ± 3.1
*t*	-0.721	-1.020	2.818	0.459	-0.816	2.318
*P*	0.472	0.309	0.005	0.647	0.416	0.022

## Data Availability

The data used to support the findings of this study are included within the article.
